# Therapeutic Effect of Electronic Endoscopic Hematoma Removal on Hypertensive Basal Ganglia Cerebral Hemorrhage Based on Smart Medical Technology

This article has been retracted.

**DOI:** 10.1155/2021/7486249

**Published:** 2021-06-08

**Authors:** Yiping Wu, Shan Zhang, Yu Dong, Xiangzhu Shen, Yafei Han, Yimeng Li, Wei Xu, Ke Ma, Huichang Tang, Dezhen Yang, Haichang Li

**Affiliations:** ^1^Neurology of Handan Central Hospital, Handan 056008, Hebei, China; ^2^Neurosurgery of Handan Central Hospital, Handan 056008, Hebei, China; ^3^Graduate School of Hebei North University, Handan 056008, Hebei, China

## Abstract

The medical and health industry has successively experienced three stages of digital medical treatment, local area network medical treatment, and internet medical treatment. With the rapid development of technologies such as the Internet of Things, big data, and artificial intelligence, emerging applications and service models have gradually penetrated into all aspects of the medical and health field. At this point, the informatization development process of the medical industry has entered the stage of smart medical treatment. (Smart medical system is a new medical system that improves users' medical experience and provides users with better services. Due to the cumbersome, complicated, and mechanically rigid environment of the past medical service, there was no uniform standard. In order to create a reliable and open medical service environment, an intelligent medical system came into being.). A diversified technical foundation and smart medical protection, conducive to providing patients with high-quality medical services, are established. This article mainly introduces the analysis of the therapeutic effect of smart medical electronic endoscopic hematoma removal on hypertensive basal ganglia cerebral hemorrhage and aims to inject advanced technology and vitality of smart medical treatment into the treatment of hypertensive basal ganglia cerebral hemorrhage by hematoma removal and help the doctor to treat the patient. This article proposes the research methods of smart medical application in the treatment of hypertensive basal ganglia cerebral hemorrhage with electronic endoscopic hematoma removal, including smart medical overview, intracranial hematoma removal for hypertensive basal ganglia cerebral hemorrhage, and smart medical bioelectric signal classification. The recognition algorithm is used to realize the smart medical application of the electronic endoscopic hematoma removal in the treatment of hypertensive cerebral hemorrhage in the basal ganglia area. The experimental results show that the removal of intracranial hematoma based on smart medicine can effectively improve the removal rate of intracranial hematoma, with a recovery rate of 26.73% and a significant efficiency of 36.49%.

## 1. Introduction

With the rapid development of information technology in the medical industry, smart medical technology has become the focus of widespread attention at home and abroad. Smart healthcare is user-centric, with medical information as the main line, using big data, Internet of Things, cloud computing, artificial intelligence, and other technologies to achieve close interaction among patients, medical staff, medical institutions, and medical equipment and establish scientific, accurate, efficient, and reasonable medical service system. Smart medical technology plays an important role in alleviating the conflicts between doctors and patients caused by information asymmetry and regional health differences caused by unreasonable allocation of medical resources and improving the level of medical services.

The smart medical treatment service system uses big data, cloud computing technology, and Internet of Things technology to establish an electronic medical record database. Paper medical records are inconvenient to store, inconvenient to carry, and easy to lose. It will cause difficulties for doctors to read and make it impossible for doctors to fully understand the patient's past medical history. A big data electronic medical record database is established so that doctors can view the patient's past disease history online and have a comprehensive understanding of the patient's physical condition and medication contraindications. The big data medical record database can also provide a wealth of pathological cases for medical research, provide sufficient data support for the occurrence, development, and prognosis of the disease, provide medical advice for disease prevention and control, and push the development of the medical industry. Now with the popularization of mobile payment methods such as Alipay and WeChat Pay, users can use mobile payment. With the payment of inspection fees and the trouble of queuing for free and cash payment, this extremely user-friendly function will also be retained in our design. At the same time, an online communication platform between doctors and patients is designed so that doctors and patients can rate each other after seeing a doctor, improving service efficiency.

Cerebral hemorrhage is a common disease among cerebrovascular diseases. Although its incidence is not as high as that of cerebral infarction, the potential recovery ability of brain function is also stronger than that of cerebral infarction, but its fatality rate is also significantly higher than that of cerebral infarction. With the improvement of living conditions, the age of onset of cerebral hemorrhage has gradually become younger, significantly reducing the quality of life of middle-aged patients, and effective treatment of cerebral hemorrhage has become a concern of most scholars. (There are two main treatment methods for hypertensive cerebral hemorrhage: one is conservative treatment, and the other is craniotomy. Minimally invasive removal between these two methods can not only remove most of the hematoma, but also avoid the major trauma to the brain caused by surgery.) The fatality rate within the first month after the onset of hypertensive intracerebral hemorrhage is 30%∼50%, and more than 30% of the survivors also have dysfunction; the fatality rate of traditional internal and surgical treatment is 46.7%∼90% and 67.9%; the recovery of nerve defect function is low. The introduction of smart medical technology into the treatment of intracranial hematoma to remove hypertensive basal ganglia cerebral hemorrhage is beneficial to improve the precision and stability of the operation and reduce the occurrence of complications. Basal ganglia hemorrhage has symptoms and signs such as putamen hemorrhage, thalamic hemorrhage, caudate nucleus hemorrhage, and serious sequelae. The study of basal ganglia hemorrhage has become one of the current medical research focuses.

From the perspective of sustainability, Hao et al. first proposed a three-dimensional evaluation model representing the original medical data, then proposed a sustainable treatment plan strategy based on the representative model, and, finally, conducted a case study on the patient's treatment plan. In the research to prove the feasibility and availability of the strategy, this method is less theoretically described, which is not conducive to reference research [1]. Zhang et al. found that the Internet of Things is rapidly spreading as a new communication paradigm, so many research studies have been conducted on various applications, especially the application of the Internet of Things in intelligent medical systems. In an intelligent medical system, many medical devices are distributed in popular areas such as stations and medical centers, and the distribution of such high-density medical devices can cause severe communication performance degradation, which is called a coexistence problem. The high cost of this research is not conducive to popularization in practice [2]. Jiang et al. believed that, with the development of medical technology based on multimedia and pattern recognition, smart medical applications in smart hospitals and personal smart medical care play an important role in our lives. He proposed an energy-saving multicast routing method in multihop wireless networks for smart medical applications. This method uses topology control and sleep mechanisms to obtain the best routing strategy with the highest network energy efficiency to construct network multicast routing. This study lacks the support of experimental data and is impractical [3].

The innovations of this paper are as follows: (1) the application of smart medical treatment in the treatment of hypertensive cerebral hemorrhage in the basal ganglia area with electronic endoscopic hematoma is proposed; (2) the application design of smart medical system is carried out.

## 2. Electronic Endoscopic Hematoma Removal in the Treatment of Hypertensive Basal Ganglia Cerebral Hemorrhage in Smart Medical Application Research Methods

### 2.1. Overview of Smart Medical Technology

Smart medical technology is the use of new ideas and new models of new generation information technologies such as the Internet of Things and cloud computing to promote the intelligentization of medical diagnosis, management, and services. Smart medical technology is an important part and important evaluation index of a smart city. At present, research on smart medicine is emerging. The implementation of smart medical technology can reduce the workload of medical staff and improve work efficiency; medical institutions can be connected with healthcare institutions, and medical information can be shared between patients and medical institutions. It can provide patients with a more scientific and effective medical service plan, which reduces the cost of medical services to a certain extent and can use data mining technology to predict diseases and provide a scientific basis for doctors' decisions [4]. The smart medical application of the Internet of Things is shown in Figure 1 (picture from ocamar.com). The current diagnostic methods are CT examination, MRI examination, DSA examination, and cerebrospinal fluid examination.

### 2.2. Intracranial Hematoma Removal for Hypertensive Cerebral Hemorrhage in the Basal Ganglia

#### 2.2.1. Pathological Basis

Hypertensive cerebral hemorrhage is a spontaneous cerebral hemorrhage caused by high blood pressure. The main pathological basis is hypertension and arteriosclerosis, in which arteriosclerosis will lead to thickening of the arterial intima and atherosclerotic plaque, making the lumen relatively narrow [5]. In addition, the elastic layer and glassy changes in the middle layer of the fibrotic arterioles can increase the fragility of the vessel wall. When blood pressure fluctuates drastically, the damaged blood vessels cannot be adjusted automatically, high blood pressure will easily rupture, or tiny aneurysms will form in the weakest part, which will cause bleeding for a long time [6, 7].

#### 2.2.2. Treatment Methods

There are two main treatment methods for hypertensive cerebral hemorrhage: one is conservative medical treatment, and the other is surgical craniotomy. Minimally invasive removal is between these two methods, which can not only remove most of the hematoma, but also avoid the large trauma to the brain caused by the surgical operation [8]. The specific implementation method is as follows: according to the position of the hematoma, choose the supine or lateral position, routine disinfection, and drape, use 2% lidocaine for local anesthesia at the puncture point, and then use an electric drill to drive the YL-1 intracranial hematoma to smash the puncture needle. After drilling through the scalp, skull, and dura in the vertical sagittal plane, withdraw the electric drill, pull out the metal needle core, insert the blunt round plastic needle core, and slowly push in [9, 10]. After reaching the surface of the hematoma, pull out the needle core, cover the cap, and connect the drainage tube to the side hole. Use a syringe to suck the liquid part of the hemorrhage surface. If resistance is encountered, the puncture needle can be rotated in situ to adjust the position of the side hole of the needle tip. Then insert the blunt round-end needle core and slowly deepen the puncture needle until the center of the hematoma [11–13]. After confirming that the puncture needle is positioned at the center of the hematoma, take out the needle core, suck slowly with a syringe, first aspirate the liquid hematoma, and then use a needle-shaped hematoma pulverizer to repeatedly flush the hematoma in equal amounts. After the flushing fluid becomes light, inject the hematoma into the hematoma cavity to liquefy. It should be rinsed 2 to 3 times a day. After the operation, the CT should be reviewed regularly according to the drainage and the condition to understand the drainage of the hematoma. The needle can be removed when the hematoma has cleared up to 85% [3, 5].

### 2.3. Smart Medical Bioelectric Signal Classification and Recognition Algorithm

#### 2.3.1. TDMA Biological Signal Acquisition

TDMA converts the time axis into a certain time element and divides each time element into time slots. In each time element, each slave node is allocated a certain number of time slots to send signals. The nodes are not sending signals when it is in a dormant state [1]. Each node in the network has a precise point in time and is synchronized with the time of the master node, thus forming a unified system clock [14]. The division of TDMA network time slots in a multinode system is determined by the physiological signals collected by the nodes, and the efficiency of the network must be considered [15]. In the TDMA protocol, the master node sends control frames to all slave nodes in turn, and then the slave node sends data and responds to the master node. The slave nodes do not communicate with each other. This compares the system's performance when transmitting a specific amount of data. For bit energy consumption [16], assuming that the total number of bits that need to be transmitted in the system is *C*, the number of system data packets *m* can be expressed as the following formula, where *S*_*ds*_ represents the unit of data frame length:

(1) $$\begin{array}{c} m=\frac{c}{8\times S_{ds}}. \end{array}$$

In the process of multinode communication, we use *S*_*tm*_ to represent the length of the polling data frame sent by the master node and *r* to represent the data throughput during human body communication [17, 18]. Then, the time *T*_*tm*_ when the master node sends the control frame has the following formula:

(2) $$\begin{array}{c} T_{tm}=\frac{S_{tm}}{r}. \end{array}$$

After receiving the request frame, the slave node responds to the master node [19]. Assuming that *S*_*cs*_ and *S*_*ds*_ are the control field and data segment in the response frame, the time *T*_*ts*_ when the slave node sends the response frame to the master node has the following formula:

(3) $$\begin{array}{c} T_{ts}=\frac{S_{ds}+S_{cs}}{r}. \end{array}$$

Assuming that the average bit error rate of the human body communication system is BER, the data packet is retransmitted in the case of packet loss [20, 21]. Then, the probability of successful system data packet transmission can be calculated as

(4) $$\begin{array}{c} p={\left(1-\text{BER}\right)}^{S_{p}\times 8}, \end{array}$$

where *S*_*p*_ is the number of bytes in the data packet during transmission [22]. Considering that the node enters the standby mode when not sending or receiving data, combined with the above formula, the energy consumed by the network to successfully transmit a data packet is

(5) $$\begin{array}{c} E_{t1}=\left[N\times \rho_{r}\times T_{tm}\times \frac{1}{p^{2}}+\rho_{t}\times T_{ts}\times \frac{1}{p}+\rho_{i\;d}\times T_{ts}\times \left(N-1\right)\right]. \end{array}$$

Among them, *N* is the number of slave nodes in the system, and *ρ*_*r*_, *ρ*_*t*_, and *ρ*_*i*  *d*_ are the received signal, transmitted signal power, and idle power of the node, respectively [23, 24]. For the master node, the energy consumed by the network to successfully transmit a data packet is

(6) $$\begin{array}{c} E_{t2}=\left[\rho_{r}\times T_{tm}\times \frac{1}{p^{2}}+\rho_{t}\times T_{ts}\times \frac{1}{p}\right]. \end{array}$$

Therefore, the total energy consumed by the system to transmit *m* data packets can be calculated as

(7) $$\begin{array}{c} E_{t}=\left(E_{t1}+E_{t2}\right)\times m. \end{array}$$

Then, the bit energy consumption of the TDMA system is

(8) $$\begin{array}{c} E_{tc}=\frac{E_{t}}{c}. \end{array}$$

#### 2.3.2. Classification of Biological Signals

Bioelectric signals such as ECG and EEG have the characteristics of strong noise, strong randomness, nonlinearity, chaos, etc. and have great variability for different individuals and scenes [25]. Research on the processing and automatic classification of these signals is the key technology and difficulty of smart medical equipment. For the classification of biological signals, support vector machine (SVM) classification of biological signal recognition algorithms can be used [26]. Support vector machine (SVM) classification is based on the principle of minimizing structural risk, seeking an optimal hyperplane, which maximizes the blank area on both sides of the hyperplane while ensuring the accuracy of the training sample classification [27, 28]. The linear discriminant function is as formula (9):

(9) $$\begin{array}{c} f\left(x\right)=\langle w,x\rangle +b. \end{array}$$

The normalized form of the equation of the optimal classification line *L* is

(10) $$\begin{array}{c} \langle w,x\rangle +b=0. \end{array}$$

The optimal classifier is as follows:

(11) $$\begin{array}{c} y_{i}\left(\langle w,x_{i}\rangle +b\right)\geq 1,\;i=1,2,\ldots ,n, \end{array}$$

(12) $$\begin{array}{c} \min J\left(w\right)=\frac{{\left\|w\right\|}^{2}}{2}. \end{array}$$

Obtained by Lagrangian function,

(13) $$\begin{array}{c} L\left(w,b,a\right)=\frac{1}{2}{\left\|w\right\|}^{2}-\overset{n}{\underset{i=1}{\sum }}a_{i}\left(y_{i}\left(wx_{i}+b\right)-1\right)a_{i}. \end{array}$$

The optimal solution *a*′=(*a*_1_′, *a*_2_′,…,*a*_*i*_′)^*h*^ is obtained [29, 30]. The modulus tools are as follows:

(14) $$\begin{array}{c} {\left\|w^{\prime }\right\|}^{2}=2w\left(a^{\prime }\right)=\sum_{SV}a_{i}^{\prime }a_{j}^{\prime }\left(x_{i}x_{j}\right)y_{i}y_{j}. \end{array}$$

The finally obtained biological signal classification function expression is

(15) $$\begin{array}{c} F\left(x\right)=\mathrm{sgn}\left(\overset{n}{\underset{SV}{\sum }}y_{i}a_{i}^{\prime }\left(x_{i}x\right)+b\right). \end{array}$$

The steps of the above method for hematoma removal are shown in Table 1.

## 3. Smart Medical Application in the Treatment of Hypertensive Intracerebral Hemorrhage in the Basal Ganglia Area with Electronic Endoscope

### 3.1. Application Design of the Smart Medical System

#### 3.1.1. Overall System Design

This article chooses the Zhiyun IoT platform provided by the laboratory as the development platform [31]. The Zhiyun platform can support the data access, classified storage, and data mining functions of a large number of terminals, and the platform uses a background analysis management system based on the B/S architecture and can support users to use WEB to manage and monitor the data center, with data storage, message push, and data analysis functions. The smart medical system is composed of collection terminals, base stations, IoT core network, NB server, smart cloud platform, hospital server, and system management software. In this system, the collection terminal has the function of collecting the patient's blood glucose level information and using the narrowband Internet of Things to send the encapsulated CoAP message to the base station; the base station and the IoT core network mainly realize the terminal access to the network and transfer the information sent by the terminal to the binding. The NB server in this system refers to the server bound to the internal NB card of the collection terminal. The server can receive the CoAP message from the collection terminal and send it to the Zhiyun server using the TCP protocol; the Zhiyun server stores the messages sent by the NB server and has the function of interacting with the system management software through the interface; the hospital server has the function of interacting with the system management software to realize the call to the system database; the system management software has the function of interacting with the Zhiyun server and the hospital server. The function realizes the processing and calling of related information.

#### 3.1.2. System Structure Design

Perception layer is mainly composed of blood glucose collection sensor, temperature sensor, and collection terminal composed of STM32F103 single-chip microcomputer and BC95 module, which realizes the collection, calculation, and information upload function of patient's blood glucose value and temperature information.

Network layer mainly realizes the long-distance and reliable transmission of information. This article mainly realizes the reliable transmission of information through communication technologies such as NB-IoT and Internet.

Platform layer provides users with the storage, access, and control functions of collected data by using cloud platform technology. This article mainly uses the third-party Zhiyun platform technology to realize the processing of sorting, storing, and accessing collected data.

Application layer mainly uses the analyzed and processed perception data to provide users with a variety of different types of services. This article implements the acquisition, processing, and use of collected information through system management software located on the PC and mobile terminals, and it provides users with different types of services.

#### 3.1.3. System Data Interaction

The data interaction process between the collection terminal and the Zhiyun platform is as follows: it is when the patient holds the collection terminal in the specified time (such as an empty stomach in the morning, 2 hours after breakfast, before lunch, two hours after lunch, two hours before dinner, and two hours after dinner) to collect blood glucose values. When sending information, the terminal will first perform the system initialization operation and then initialize the NB-IoT communication module to enable it to access the network. After the network access is successful, the CoAP protocol is used to send the ID and KEY of the Zhiyun platform to the NB server to request authentication, and the NB server receives it. After that, the payload part of the CoAP message will be extracted first and then sent to the Zhiyun platform using the TCP protocol. After receiving the message, the Zhiyun platform will authenticate the ID and KEY. After the authentication is successful, the patient can insert the blood glucose meter test strip into the terminal. The terminal is triggered to collect blood glucose concentration and temperature information, and then the terminal will control the display module to output the calculated blood glucose concentration and time information. Then the terminal can encapsulate and send the blood glucose concentration and NB card information according to the agreed communication protocol format. After the server receives the message, it unpacks the message, sends back an ACK response message to the terminal, and then uses the TCP protocol to send the content of the message to the Zhiyun platform. After receiving the TCP message, the Zhiyun platform will send the information to the terminal according to the terminal address. The sent information and the time of receiving terminal information are stored in the database.

### 3.2. System Software Technology Selection

The software technology used by the system includes a server with JavaWeb as the core and browser and mobile programs with JavaScript, HTML, and CSS as the core. The database uses SQLite database.

#### 3.2.1. JavaWeb

JavaWeb is an enduring hot technology in the Web field, and it is the collective name for a series of technologies that use the Java language platform. Both classic and reliable enterprise-level or lightweight JavaEE systems are widely used in software development. In addition, there are two other architectures that are also widely used: .Net and PHP. The original Taobao used the PHP system, and Jingdong used the .Net system. However, with the rapid development of the Internet, the business scale of the e-commerce platform has become larger and larger. In order to adapt to high concurrency and higher stability, it will take the lead in the competition. Major e-commerce platforms have been changed to JavaWeb technology architecture. The JavaWeb architecture can be refined into the following five-layer structure.

1. Presentation layer interacts with users. Usually composed of JSP pages, the presentation layer collects the user's request and returns the business result to the user.
2. Controller layer is composed of controllers in the MVC architecture. After intercepting the request, the method of the business logic layer is called to process the request, and the result of the request is forwarded to the corresponding presentation layer component.
3. Business logic layer implements business logic methods and generates and processes logic data.
4. Data access object layer is referred to as DAO layer for short. It achieves atomic operations on the database.
5. Domain object layer of the system is composed of a series of simple Java objects.

#### 3.2.2. Database Technology

SQLite is lightweight cross-platform database software based on the SQL language. It is also an ACID-compliant relational database management system. Compared with the scalability, concurrency, centralization, and cluster control of MySQL, Oracle, PostgreSQL, and other B/S system databases, SQL emphasizes economy, efficiency, reliability, and simplicity. It has the advantages of high query and storage efficiency, support for simultaneous access of multiple processes, small running memory, and single file storage of database content. It is used to establish contact with various databases, operate and process data, and complete addition, deletion, modification, and query operations.

The steps of hematoma removal are shown in Table 2.

## 4. Objective to Analyze the Therapeutic Effect of Electronic Endoscopic Hematoma Evacuation on Hypertensive Basal Ganglia Hemorrhage Based on Smart Medical Technology

### 4.1. System Performance Analysis

In the previous article, this article elaborated the key technologies, overall system design, software, and structure design methods of the smart medical system in detail (The analysis part of the article first explained the module performance of the system, carried out various tests, and then applied it to the study of the specific problem of cerebral hemorrhage and illustrated the chart.). In addition, in order to ensure the normal operation of the system, this section will test the performance of each module of the system and conduct targeted tests in terms of NB-IoT wireless communication performance, data collection accuracy, and multiterminal management. This article will simulate the normal working environment to test the system and build the software and hardware environment according to the test requirements. The hardware environment includes a laptop computer (simulating hospital server, WIN10 32-bit operating system), a digital multimeter, and NB-IoT communication. There are five modules and five smart medical terminals developed by this system; the software environment is the smart medical platform software, SQLite database, and smart cloud platform developed by this system.

1. In order to enable the smart medical system to work stably in long-distance scenarios, the system conducts independent tests on the NB-IoT wireless communication performance. On the one hand, under certain experimental conditions, the transmission distance and packet loss rate of the NB-IoT module can be tested in an open and unobstructed area; on the other hand, the transmission distance and packet loss rate of the NB-IoT module can be tested indoors under the same experimental conditions rate. The nominal transmission distance of this module is up to 2000 meters. In this paper, the communication performance of the NB-IoT module is tested at equal intervals within a distance of 400 meters to 2000 meters in a straight line, and 1500 packets are sent for each test. The outdoor measured data of the communication performance of the NB-IoT module are shown in Table 3 and Figure 2.
2. As shown in the chart, when the communication distance is within 400 meters, no packet loss can be guaranteed, the communication distance exceeds 400 meters, and the communication performance gradually decreases; the average packet loss rate between 400 meters and 2000 meters reaches 7.60%.
3. The transmission distance and packet loss rate of the NB-IoT module were tested indoors under the same experimental conditions. This article tested the communication performance of the NB-IoT module at equal intervals from the third floor to the tenth floor of the building. The indoor measured data of the communication performance of the NB-IoT module with 1500 packets sent in this test are shown in Table 4 and Figure 3.
4. As shown in the data in the chart, when the communication distance is below the third floor, no packet loss can be guaranteed. As the third floor goes up, the communication performance gradually decreases; the average packet loss rate between the third floor and the tenth floor reaches 2.67%.
5. When the system collects signals, the classification accuracy is an important indicator. Therefore, the smart medical system needs to have strict requirements on the accuracy of data classification. This article has made a test to verify the accuracy of data classification. At the same time, it also evaluates the classification accuracy of the algorithm in this paper in conjunction with a long-running experiment such as system performance testing. The specific situation is shown in Table 5 and Figure 4.

Through analysis, it can be obtained that the classification accuracy of the system data of the six tests is 97.14%, and the algorithm classification accuracy rate is relatively high. It can better serve the smart medical signal collection and classification, which is helpful for smart medical treatment in electronic endoscopic hematoma removal, used in the treatment of hypertensive intracerebral hemorrhage in the basal ganglia.

### 4.2. Efficacy Analysis

1. After treatment, the amount of residual hematoma in the hematoma removal treatment group and the conservative treatment group showed a significant downward trend. Compared with the conservative group, the surgical group had an advantage in the amount of residual hematoma at one, two, four, six, and eight days after surgery. The results are shown in Table 6 and Figure 5.
2. The treatment of cerebral hemorrhage in our country mainly includes conservative treatment and surgical treatment. Regardless of whether it is conservative treatment or surgical treatment, the treatment goals are focused on clearing hematomas and reducing intracranial pressure by removing intracranial hematoma, reducing the space-occupying effect of intracranial hematoma, maximizing the recovery of compressed nerve cells, improving the patient's neurological impairment, and providing more space and possibility for patient recovery to prevent hematoma and the toxic damage of metabolites and transmitters to peripheral cerebral ischemic cells.
3. The treatment effects on patients in the surgical group and the conservative group are shown in Table 7 and Figure 6.

The mortality and disability rates of hypertensive basal ganglia cerebral hemorrhage are very high. (Putamen and thalamus are the two most common sites of hypertensive intracerebral hemorrhage. Typical signs of triple sign (contralateral hemiplegia, hemisensory loss, hemianopia, etc.) can be seen. Massive hemorrhage can cause disturbance of consciousness or can penetrate the brain tissue into the ventricle and appear in bloody CSF. It is not common to directly penetrate the cortex.) Conservative medical treatment is effective for small hemorrhage, but it is powerless for massive hemorrhage. The value of surgical treatment of cerebral hemorrhage cannot be confirmed at present, and one is urgently needed. It can quickly remove hematoma and small trauma. The removal of intracranial hematoma based on smart medicine can effectively improve the clearance rate of intracranial hematoma, shorten the time taken to remove hematoma, improve the removal efficiency of intracranial hematoma, effectively improve the patient's serum hs-CRP level, and avoid intracranial infection. The recovery rate reaches 26.73%, and the apparent efficiency reaches 36.49%, which improves the effect of clinical treatment. At the same time, in the long run, it has clinical value for improving the quality of life of patients after surgery and ensuring that patients get a good prognosis.

## 5. Conclusions

Smart healthcare expands the channels for users to obtain medical information, and patients achieve health management goals through information interaction with medical staff, medical institutions, and smart devices. Based on the purpose of helping medical staff and serving patients, this article takes the application of smart medicine to the treatment of hypertensive basal ganglia cerebral hemorrhage with electronic endoscopic hematoma removal as the research object and uses a combination of theoretical analysis and empirical research to try to carry out electronic endoscopic hematoma removal for the application of smart medicine in the treatment of hypertensive basal ganglia cerebral hemorrhage. It also tries to conduct in-depth analysis and research on the effect of electronic endoscopic hematoma removal on hypertensive basal ganglia cerebral hemorrhage combined with smart medical treatment. Due to the limitations of time and academic level, this article has some limitations and deficiencies, and there is still academic space that needs to be explored and improved. For example, the algorithm has not been simplified, and the research content is not convenient for promotion and use. In future research, the algorithm will be optimized for the promotion of the research content.

## Figures and Tables

**Figure 1:** Smart medical applications of the IoT.

**Figure 2:** Outdoor test results.

**Figure 3:** Indoor test results.

**Figure 4:** Algorithm classification accuracy.

**Figure 5:** Average residual amount of hematoma in patients (mg/L).

**Figure 6:** Treatment effects.

**Table 1:** Part of the technical process of the method in this article.

Electronic endoscopic hematoma removal in the treatment of hypertensive basal ganglia cerebral hemorrhage in smart medical application research methods	2.1	Overview of smart medical		
	2.2	Intracranial hematoma removal for hypertensive cerebral hemorrhage in the basal ganglia	1	Pathological basis
			2	Treatment
	2.3	Smart medical bioelectric signal classification and recognition algorithm	1	TDMA biosignal acquisition
			2	Biosignal classification

**Table 2:** Some steps of the experiment in this article.

Smart medical application of electronic endoscopic hematoma clearing hypertensive basal ganglia cerebral hemorrhage			
3.1	Application design of smart medical system	3.2	System software technology selection
1	Overall system design	1	JavaWeb
2	System structure design	2	Database technology
3	System data interaction		

**Table 3:** Outdoor test results.

Test distance (meter)	Number of received packets	Number of packets not received	Packet loss rate (%)
400	1500	0	0.00
500	1491	9	0.60
900	1412	88	5.87
1300	1374	126	8.40
1700	1309	191	12.73
2000	1227	273	18.20
Average	1386	114	7.60

**Table 4:** Indoor test results.

Floor	Number of received packets	Number of packets not received	Packet loss rate (%)
Third floor	1500	0	0
Fourth floor	1494	6	0.40
Fifth floor	1481	19	1.27
Sixth floor	1464	36	2.40
Seventh floor	1452	48	3.20
Eighth floor	1438	62	4.13
Ninth floor	1429	71	4.73
Tenth floor	1420	80	5.33
Average	1460	40	2.67

**Table 5:** Algorithm classification accuracy.

Experiment number	Algorithm classification accuracy (%)
1	96.42
2	97.31
3	95.76
4	97.14
5	98.06
6	98.14
Average	97.14

**Table 6:** Average residual amount of hematoma in patients (mg/L).

Time	Operation group	Conservative group
1 d after surgery	18.61	21.58
2 d after surgery	18.24	21.12
4 d after surgery	16.76	20.07
6 d after surgery	14.42	18.65
8 d after surgery	12.09	15.17

**Table 7:** Treatment effects.

Curative effects	Operation group (%)	Conservative group (%)
Cure rate	26.73	22.17
Apparent efficiency	36.49	29.53
Efficiency	28.64	28.14
Inefficiency	6.56	16.42
Fatality rate	1.58	3.74

## Data Availability

No data were used to support this study. Data sharing is not applicable to this article as no datasets were generated or analyzed during the current study.
